# Long non-coding RNA FENDRR inhibits migration and invasion of cutaneous malignant melanoma cells

**DOI:** 10.1042/BSR20191194

**Published:** 2020-03-18

**Authors:** Xu-e Chen, Pu Chen, Shanshan Chen, Jin Lu, Ting Ma, Guang Shi, Liang Sheng

**Affiliations:** 1 Department of Dermatology, Guizhou Provincial People’s Hospital, Guiyang, Guizhou 550002, China; 2 Department of Information, Guizhou Province Hospital of Traditional Chinese Medicine, Guiyang, Guizhou 550001, China

**Keywords:** FENDRR, invasion, JNK/c-Jun pathway, Malignant melanoma, migration, MMP2/MMP9

## Abstract

The present study aimed to investigate the effects of lncRNA FENDRR on the migration and invasion of malignant melanoma (MM) cells. The expression levels of FENDRR in MM tissues and MM cell lines were detected using qRT-PCR, followed by construction of FENDRR-knocked down and overexpressed stable cells. Then the effects of FENDRR on cell proliferation, migration and invasion were detected using MTT assay and Transwell assay. The protein expression levels of matrix metallopeptidase 2 (MMP2), MMP9, and related factors in JNK/c-Jun pathway were detected using Western blot. FENDRR was down-regulated in MM tissues and cell lines. Besides, its expression levels in different MM cells were diverse. Knockdown of FENDRR facilitated MM cells proliferation, migration and invasion in A375 cells, while overexpressing FENDRR had reverse results. In addition, MMPs and JNK/c-Jun pathway involved in the FENDRR-mediated regulation of MM cell proliferation, migration and invasion. Our results demonstrated that FENDRR mediated the metastasis phenotype of MM cells by inhibiting the expressions of MMP2 and MMP9 and antagonizing the JNK/c-Jun pathway.

## Introduction

Malignant melanoma (MM) is a highly aggressive skin cancer, which develops from melanocytes [1]. The incidence of MM is rising more rapidly than any other prevalent cancers [2]. MM accounts for the vast majority of skin cancer patient deaths [3]. MM has proclivity to metastasize, and patients with metastatic MM has a poor prognosis [4]. The patients who are diagnosed as MM early usually have high 5-year survival rates, but patients with metastatic MM has a 5-year survival rate of only 5–10% [5]. Currently, the therapeutic options to MM that have metastasized and invaded into the dermis are very limited. Therefore, a better understanding of the etiologies and genetic underpinnings of MM is critical for the development of therapeutic strategies in this malignancy.

Long noncoding RNAs (lncRNAs), a group of RNA molecules with more than 200 nucleotides, have been revealed to play key roles in numerous biological processes and contribute toward the etiology of disease, especially neoplasm [6,7]. As a result, lncRNAs are emerging as regulators of cancer progression and have the potential to be used as key diagnostic and therapeutic markers [8]. Importantly, a large number of lncRNAs have been identified to be misexpressed in MM, such as lncRNA MALAT1 and lncRNA HOTAIR [9,10]. Additionally, several lncRNAs, like lncRNA SAMMSON and lncRNA CASC15, have been reported as putative modulators for melanoma proliferation, survival and metastatic behaviors [11]. LncRNA FENDRR is essential for the development of heart and body wall, which has recently been found to play an important role in the development and metastasis of gastric cancer [12]. However, its clinical role in MM remains yet to be found.

In the present study, we intended to investigate the expression levels of FENDRR in MM from molecular point of view and then to elucidate the relationships between its dysregulation and cell proliferation, metastasis and invasion. We focused on the underlying molecular mechanism of FENDRR affecting MM in order to provide new insight into the treatment of this disease.

## Materials and methods

### Tissue samples

A total of 90 paraffin-embedded samples, including 30 cases of cutaneous malignant melanoma with metastasis (M1), 30 cases of cutaneous malignant melanoma without metastasis, and 30 cases of pigmented nevus, were collected from 2010 to 2014 in the Department of Pathology of Dermatology, Guizhou Provincial People’s Hospital. In addition, 30 normal skin samples obtained from orthopedic surgery were used as controls. These participants were aged between 22 and 76 years old, with an average age of 58.8 ± 9.2 years.

All patients had provided their informed consent before the study. Total procedures in this study were approved by our hospital’s protection of human ethics committee.

### Cell culture, treatment and transfection

Hacat, A375, SK-Mel-28, and SK-Mel-110 cell lines were obtained from American Type Culture Collection, U.S.A. These cells were cultured in Dulbecco’s Modified Eagle’s Medium (DMEM) (Thermo Fisher Scientific, U.S.A.) with 10% fetal bovine serum (FBS) (Hyclone, U.S.A.), 100 μg/ml streptomycin, and 100 U/ml penicillin (Thermo Fisher Scientific) in a humidified incubator at 37°C in 5% CO_2_. Cells were digested with trypsin (Sigma Aldrich Co., U.S.A.) when they reached 70–80% confluence.

Before cell transfection, 20 μmol/l SP600125 (JNK inhibitor) was added into cells and incubated for 12 h.

Lentivirus was made to generate A375-FENDRR-si and SK-Mel-110-FENDRR- overexpressing cell lines. A shRNA with high FENDRR knockdown efficiency was used. Total 15 μg pGag/pol, 10 μg pVSVG, and 20 μg pSIREN-RetroQ-ZsGreen1-FENDRRshRNA plasmid were co-transfected into sub confluent 293T cells using Lipofectamine® 2000 Reagent (Thermo Fisher Scientific). After 72 h, the viral supernatants were collected, and the pLVX-TRE3G-ZsGreen1 vector harboring the FENDRR cDNA lentivirus was harvested as well. Subconfluent A375 cells were then infected with harvested lentivirus. Individual colonies of stable overexpression of FENDRR and control colonies were isolated.

### MTT assay

After transfection, cells were seeded into 96-well culture plates with 5000 cells/well and cultured in a humidified incubator at 37°C and 5% CO_2_ for 24, 48 and 72 h, respectively. Then 20 μl of 5 mg/ml thiazolyl blue tetrazolium bromide (MTT) (Amresco, U.S.A.) was added for another 3 h incubation in a humidified atmosphere containing 5% CO_2_ at 37°C. Subsequently, cells were harvested in 150 μl dimethylsulfoxide (DMSO) (Amresco, U.S.A.) and shaken for 10 min. Finally, cell lysate was analyzed for MTT activity to indicate cell viability by determining absorbance at 492 nm.

### Clonogenic assay

After transfection, cells were plated into 60 mm tissue culture dishes at a density of 200 cells/dish. Cells were then grown in RPMI-1640 medium containing 10% FBS for 14 days. Then cells were fixed and stained with Diff-Quick, followed with air dry. The colonies were counted under microscope (IX83, Olympus, Japan), and cell number of each colony was at least 30 cells.

### Cell migration and invasion assays

For the migration assay, 5 × 10^4^ cells in serum-free media were added to the upper chamber of an insert (Millipore, U.S.A.) after 48 h of transfection. For the invasion assay, 1 × 10^5^ cells in serum-free medium were seeded into the upper chamber of an insert coated with Matrigel (Sigma Aldrich Co., U.S.A.). The lower chamber was enveloped with DMEM containing 10% FBS. After 24 h of incubation, the cells were removed with cotton wool, and cells that had migrated or invaded through the membrane were stained with 0.1% Crystal Violet. Finally, cells were imaged and counted using an IX71 inverted microscope (Olympus, Japan).

### Quantitative real-time polymerase chain reaction (qRT-PCR)

Total RNAs were extracted from tissues or cells using Trizol reagent (Invitrogen, U.S.A.). The expressions of FENDRR in tissues and cells were evaluated using qRT-PCR kits (Takara, Dalian, China). The primers were FENDRR (forward, 5′-TAAAATTGCAGATCCTCCG-3′, and reverse, 5′-AACGTTCGCATTGGTTTA GC-3′), and GAPDH (forward, 5′-GGGCATCTTGGGCTACAC-3′, and reverse, 5′-GGTCCAGGGTTTCTTACTCC-3′). The relative expression of FENDRR was calculated using the comparative cycle threshold (CT) (2^−ΔΔCT^) method. Glyceraldehyde-3-phosphate dehydrogenase (GAPDH) was used as the endogenous control.

### Western blot assay

The transfected cells were lapped with RIPA lysis and extraction buffer (Sangon Biotech, Shanghai, China). The protein concentration was detected using a BCA protein assay kit (Pierce, U.S.A.). The protein (20 μg) was subjected to a 10% sodium dodecylsulfate-polyacrylamide gel electrophoresis (SDS-PAGE) and transferred to polyvinylidene fluoride (PVDF) membrane (Sigma, U.S.A.). Then the membranes were incubated with primary antibodies (matrix metallopeptidase 2 (MMP2), MMP9, c-Jun N-terminal kinase (JNK), p-JNK, c-Jun, p-c-Jun; 1:1000 dilution) at 4°C overnight, followed by incubation with horseradish peroxidase labeled secondary antibody (1:1000 dilution) for 1 h at room temperature. The bands were visualized using electrochemiluminescence (ECL) chromogenic substrate. The intensity of the bands was quantified by densitometry. GAPDH was served as the internal control.

### Statistical analysis

All data were expressed as mean ± standard deviation (SD), and the difference among all groups was compared by one-way analysis of variance. *P*-value < 0.05 was considered to be statistical significant. All the statistical analyses were carried out by SPSS 21.0 (IBM Corporation, Armonk, NY U.S.A.).

## Results

### Expression of FENDRR in tissues and cells

In order to investigate the expression level of FENDRR in different tissue samples and cell lines, qRT-PCR was performed. Our results showed that among the four kinds of tissues, FENDRR had the lowest expression levels in MM with metastasis, followed by MM without metastasis. FENDRR had the highest expression levels in normal tissues (Figure 1A). The results suggested that FENDRR may be associated with the metastatic capability of MM. In addition, compared with normal skin cell line, FENDRR expression varied among the other three melanoma cell lines. Notably, the highest FENDRR expression levels were found in A375 cells among three melanoma cell lines, while the lowest FENDRR expression were found in SK-Mel-110 cell lines (Figure 1B). Therefore, further experiments were performed using A375 and SK-Mel-110 cells.

**Figure 1:** The expression levels of FENDRR in malignant melanoma tissues and different melanoma cells detected by qRT-PCR All experiments were repeated three times with the same sample. *: *P*<0.05, **: *P*<0.01 compared with control.

### Effect of FENDRR on cell proliferation

In order to evaluate the role of FENDRR in cell proliferation, MTT, qRT-PCR and colony formation assay were performed. FENDRR was knocked down by transfecting shRNA-FENDRR into A375 cell line and was overexpressed by transfecting pcDNA-FENDRR vector into SK-Mel-110 cell line. The expressions of FENDRR in cells after transfection were confirmed by qRT-PCR (Figure 2A). As shown in Figure 2B, the cell viability was significantly increased from 24 h after FENDRR knockdown in A375 cell line (*P* < 0.05). Whereas, FENDRR overexpression significantly reduced cell viability in SK-Mel-110 cell line (*P* < 0.05). Moreover, colony formation assay showed significant proliferative effects of FENDRR in either A375 or SK-Mel-110 cell line (Figure 2C,D). In a word, those results suggested that FENDRR had a proliferative effect on cells.

**Figure 2:** Effect of FENDRR expression on cell viability and proliferation (**A**) The expression of FENDRR in malignant melanoma cells after FENDRR knockdown and overexpression; (**B**) The viability of A375 and SK-Mel-110 cells after cell transfection detected by MTT assays. (**C** and** D**) The colony number of A375 and SK-Mel-110 cells after cell transfection detected by colony formation. All experiments were repeated three times with the same sample. *: *P*<0.05, **: *P*<0.01 compared with control.

### Effect of FENDRR on cell migration and invasion

In order to investigate the effect of FENDRR on cell migration and invasion, we performed transwell assay. As shown in Figure 3A,B, after knockdown of FENDRR in A375 cells, migration and invasion of A375 cells were significantly increased in comparison with control groups (*P*<0.05). When FENDRR were overexpressed in SK-Mel-110 cells, migration and invasion of SK-Mel-110 cells exhibited a notably decrease than those in controls (*P*<0.01). These findings indicated that FENDRR may be closely associated with migration and invasion of MM cell lines.

**Figure 3:** The changes in the (**A**) migratory and (**B**) invasive abilities of malignant melanoma cells detected by Transwell assays All experiments were repeated three times with the same sample. *: *P*<0.05, **: *P* <0.01, ***: *P*<0.001 compared with control.

### MMPs and JNK/c-Jun pathway involved in the FENDRR-mediated regulation of MM cell proliferation and metastasis

The proliferation and invasion of malignant melanoma cells involve the degradation and recombination of extracellular matrix by the activation of multiple matrix metalloproteinases (MMPs) [13]. It has been reported that antisense LncRNA FENDRR promotes migration and invasion of osteosarcoma cells through the FOXF1/MMP-2/-9 pathway [14]. To further explore the molecular mechanisms by which FENDRR contributed to the proliferation and metastasis of MM cells, we detected the protein expression levels of MMP2 and MMP9 by Western blot. The results revealed that silenced FENDRR significantly up-regulated the protein expressions of MMP2 and MMP9 in A375 cells (*P* < 0.01), whereas overexpression of FENDRR significantly decreased their expressions in SK-Mel-110 cells (*P*<0.05) (Figure 4A).

**Figure 4:** FENDRR regulated the protein expression levels of MMP2/MMP9 and JNK/c-Jun pathway (**A**) The protein expression levels of MMP2/MMP9, JNK and c-Jun after cell transfection detected by Western blot. (**B** and **C**) The changes in the (B) migratory and (C) invasive abilities of malignant melanoma cells after cells were treated with JNK inhibitor of SP600125. All experiments were repeated three times with the same sample. *: *P*<0.05, **: *P*<0.01, ***: *P*<0.001 compared with control.

Study has reported that JNK/c-Jun pathway could regulate the expressions of MMP2 and MMP9, and involves in the migration and invasion of MM [15,16]. Therefore, we investigated the protein expressions of JNK, c-Jun and their phosphorylation levels. As shown in Figure 4A, knockdown of FENDRR significantly increased the phosphorylation levels of JNK and c-Jun in A375 cells (*P* < 0.001). However, SP600125 (JNK inhibitor) treatment inhibited the effect of FENDRR knockdown (*P* < 0.01). At the same time, SP600125 also decreased the protein expressions of MMP2 and MMP9 in A375 cells with FENDRR knockdown (*P* < 0.01). Moreover, in SK-Mel-110 cells, overexpressed FENDRR significantly reduced the phosphorylation levels of JNK and c-Jun (*P* < 0.001). These results suggested that FENDER could inhibit the activation of JNK/c-Jun pathway and the expressions of MMP2 and MMP9.

To further demonstrate that JNK/c-Jun pathway involved in the migration and invasion of MM cells, we investigated the effect of SP600125 on the migration and invasion of A375 cells with FENDRR knockdown. The results showed that SP600125 treatment significantly decreased the migration and invasion of A375 cells with FENDRR knockdown (*P* < 0.05) (Figure 4B,C). Taken together, those results suggested that FENDRR had a regulating effect on MM cells through MMPs and JNK/c-Jun pathway.

## Discussion

The present study investigated the expression of FENDRR in MM tissues and cell lines and revealed that FENDRR was down-regulated in MM tissues and cell lines. Besides, its expression levels in different MM cells were diverse. Then we investigated the effect of FENDRR on cell proliferation, migration and invasion by knocking out FENDRR in A375 cell lines with abundant FENDRR expression and overexpressing FENDRR in sk-mel-110 cell lines with the least FENDRR expression. The results revealed that knockdown of FENDRR facilitated MM cells proliferation, migration and invasion in A375 cells, while overexpressing FENDRR showed reverse results. Further study found that FENDRR may regulate MM cell proliferation, migration and invasion through MMPs and JNK/c-Jun pathway.

FENDRR is first identified by Khalil et al. [17], which plays critical roles in the control of chromatin structure and gene activity by binding to polycomb repressive complex 2 (PRC2) and Trithorax group/MLL protein complexes (TrxG/MLL) [18]. Subsequent study found that FENDRR was essential for proper heart and body wall development [19]. Recently, low FENDRR expression was demonstrated to be implicated with an aggressive tumor phenotype in gastric cancer [12]. In our study, we also detected the expression of FENDRR in MM tissues and cell lines by qRT-PCR assay. Our study suggested that FENDRR was down-regulated in MM tissues and cell lines. Therefore, FENDRR may play a significant role in tumor biology in MM.

It is well known that early stages of most cancers are marked by excessive proliferation [20], while metastasis is the leading lethal cause of many cancers [21,22]. We thereby focused our investigation on the effects of FENDRR on MM proliferation, migration and invasion. The results revealed that knockdown of FENDRR significantly promoted MM cells proliferation, migration and invasion, whereas overexpression of FENDRR significantly inhibited these capacities. Those results were in line the effects of FENDRR on gastric cancer [12]. Taken together, these results suggested that FENDRR may affect the progression of MM by affecting cell proliferation, migration and invasion.

In order to explore the underlying molecular mechanism through which FENDRR contributed to cell proliferation, migration and invasion in MM, we investigated the expression levels of potential target proteins and pathway. Previous studies have demonstrated that aberrant expression of MMPs was associated with tumor initiation, development, migration and invasion in many cancers, such as lung cancer, breast cancer and hepatocarcinoma [23–25]. Specially, MMP2 and MMP9 have been reported to be closely related to the migration and invasion among numerous cancers including melanoma [26–28]. In the present study, we unraveled a significant increase in the expression levels of MMP2 and MMP9 in A375-FENDRRsi MM cells and a marked decrease upon FENDRR overexpression in SK-Mel-110 cells. Those results indicated that FENDRR may negatively regulate the expressions of MMP2 and MMP9 to involve in the migration and invasion of MM cells.

Accumulating evidence indicates that the activate JNK performs vital role in cell migration and invasion [29]. JNK belongs to the mitogen-activated protein kinase (MAPK) family. Phosphorylated JNK rapidly phosphorylates Ser-63 and Ser-73 of the c-Jun amino terminus, resulting in induction of c-Jun synthesis [30]. It has been reported that activation of JNK promotes motility and proliferation of tumor cells [31,32]. In addition, Zhou et al. [33] found that the cooperation of JNK with c-Jun played a crucial role in overexpression of Fyn related kinase-induced cell migration and invasion inhibition in glioma cells. In the present study, we determined the expression of JNK, c-Jun and their phosphorylation levels, and found that knockdown of FENDRR significantly increased the phosphorylation levels of JNK and c-Jun, whereas overexpressed FENDRR significantly reduced the phosphorylation levels of JNK and c-Jun. Furthermore, JNK inhibitor, SP600125, could decrease the expressions of MMP2 and MMP9, as well as decrease the migration and invasion of A375 cells with FENDRR knockdown. These results suggested that FENDRR may regulate cell proliferation, migration and invasion by antagonizing the JNK/c-Jun pathway in MM.

In conclusion, our study suggested that FENDRR was down-regulated in MM tissues and cell lines and the low expression of FENDRR was associated with MM cell proliferation, migration and invasion. Moreover, our results also demonstrated that FENDRR mediated the metastasis phenotype of MM cells by inhibiting the expressions of MMP2 and MMP9 and antagonizing the JNK/c-Jun pathway. Further insights into the functional implications of FENDRR may help to the treatment of MM.

## Abbreviations

DMEM: Dulbecco’s Modified Eagle’s Medium
FBS: fetal bovine serum
lncRNA: long noncoding RNA
MM: malignant melanoma
MMP: matrix metallopeptidase
